# Antibacterial and Anticancer Potentials of Presynthesized Photosensitive *Plectranthus cylindraceus* Oil/TiO_2_/Polyethylene Glycol Polymeric Bionanocomposite

**DOI:** 10.1155/2021/5562206

**Published:** 2021-10-31

**Authors:** Musarat Amina, Nawal M. Al Musayeib, Nawal A. Alarfaj, Maha F. El-Tohamy, Gadah A. Al-Hamoud

**Affiliations:** ^1^Department of Pharmacognosy, Pharmacy College, King Saud University, Riyadh 11451, Saudi Arabia; ^2^Department of Chemistry, College of Science, King Saud University, P.O. Box 22452, Riyadh 11451, Saudi Arabia

## Abstract

The present study is concerned with the fabrication of the bifunctional *Plectranthus cylindraceus* oil/TiO_2_/polyethylene glycol polymeric film for antibacterial and anticancer activities. The suggested film is based on the utility of naturally extracted *P. cylindraceus* oil in the formation of the polymeric bionanocomposite film decorated with TiO_2_ nanoparticles. The bionanocomposite film was fabricated by incorporating 15 w% of *P. cylindraceus* oil with 10 w% polyethylene glycol and 5 w% TiO_2_ nanoparticles. The active components of *P. cylindraceus* oil were verified using gas chromatography coupled with mass spectrometry (GC-MS). The surface morphology of the resulted bionanocomposite film was characterized by various spectroscopic and microscopic techniques. The antibacterial potential of the fabricated bionanocomposite film was investigated against four pathogenic strains. The obtained results revealed excellent sensitivity against the bacterial strains, particularly *E. coli* and *S. aureus*, with minimum inhibitory concentration 320 *µ*g mL^−1^ and minimum bactericidal concentration 640 and 1280 *µ*g mL^−1^ for *E. coli and S. aureus,* respectively. Polymeric bionanocomposite exerted significant cytotoxicity against human lung carcinoma cell lines in a concentration-dependent manner with an IC_50_ value of 42.7 ± 0.25 *μ*g mL^−1^. Safety assessment test against peripheral blood mononuclear cells (PBMCs) demonstrated that the bionanocomposite is nontoxic in nature. Bionanocomposite also showed potent photocatalytic effects. Overall, the results concluded that the bionanocomposite has expressed scope for multifaceted biomedical applications.

## 1. Introduction

Nanocomposites provide attractive and cost-effective thin layers with superior features for biomedical and microelectronic applications. In recent times, nanocomposites synthesized from natural biopolymers or biological resources have attained much attention. The biodegradable polymers in combination with noble metal nanoparticles offer bionanocomposites with exceptional biomedical and environmental applications [1–3]. These bionanocomposites are potentially biodegradable and versatile, and their polymeric derivatives can be prepared from a range of renewable resources such as hydrocarbon- and oxygen-rich monomers [4, 5]. Recently, the best approach for upgradation of polymers is the formation of polymeric bionanocomposites, which enhance their scope of applications. The incorporation of nanosized inorganic metallic elements in the polymers dramatically enhanced the physicochemical, mechanical, electrical, thermal features, gas barrier property, stiffness, electrical conductivity, and dimensional stability in comparison to normal polymers or conventional composites [6]. Bionanocomposites are made up of a natural polymeric matrix, renewable resources obtained from the polymer matrix, and organic/inorganic components with one or more dimensions on the nanometer scale [7]. The bionanocomposites are derived from several natural polymeric resources such as starch, cellulose, chitosan, polylactic acid, and essential oil derivatives [8–13]. Among natural resources, plant-derived essential oils have been identified as an outstanding natural biomaterial with extraordinary bioactivity, biocompatibility, biodegradability, and nontoxicity containing multifunctional groups [14, 15].

Polyethylene glycol (PEG) is an extensive antifouling hydrophilic polymer with various biomedical and industrial applications [16, 17]. The introduction of new functionalities by surface coating of PEG on different nanoparticles, proteins, and substrates enhances the biocompatibility of the host materials. Surfaces coated with PEG are well described for their antifouling ability to restrict protein adsorption, microbial attachment, and cell adhesion [18]. The antifouling property of PEG and PEG-conjugated proteins can also lower the external immune response, increase blood circulation time, and enhance the proteolytic, mechanical, and thermal stability [19]. The performances of the sustainable resources-derived polymers are further improved by the addition of different conventional nanofillers, including calcium carbonate, clays, talc, kaolin, fumed silica glass fibers carbon nanotubes, noble metal, and metal oxides [20, 21]. The resultant biocomposite unites the benefits of low-dimensional layers with a vast surface area of nanoparticles, leading to diverse useful applications in the biomedical science and the manufacturing industry.

Among various metal and metal oxides, titanium oxide nanoparticles possess unique features and interesting biological properties. Titanium oxide (TiO_2_) easily combines with the polymers, relatively stable and strong with respect to both physical and chemical properties. It is an important semiconducting material with a crystalline structure and displayed remarkable applications, including photocatalysis, solar energy conversion and field emission emitters, environmental pollution control, chemical inertness, excellent mechanical properties, nontoxicity, high refractive index, low cost, high-temperature superconductors, gas sensors, batteries, strong oxidizing power, high hydrophilicity, intense UV absorption, and strong antibacterial activity against numerous pathogens, including bacteria, fungi, algae and virus [22]. It has been frequently used in food, food packaging, cosmetics, optical devices, paints, coatings, and specifically antimicrobials due to their strong effects towards photocatalytic disinfection [23]. TiO_2_ exists in anatase (tetragonal), rutile (tetragonal), and brookite (orthorhombic) crystalline polymorphs. Rutile is the most stable form and possesses good scattering effects and has been extensively used in pigments to protect the materials from hazardous UV light [24]. In recent times, the use of TiO_2_ nanoparticles in photodynamic therapies has been constantly increasing. TiO_2_ nanoparticles and their composites and hybrids with other molecules are frequently used in the photodynamic inactivation of bacteria resistant to antibiotics and photosensitizing agents in cancer treatments [25]. TiO_2_ nanoparticles were employed as inter alia in the formation of bioconjugates with specific-cell monoclonal antibodies for malignant tumor therapies or synthesis of black TiO_2_ nanoparticles for the antimicrobial therapy against antibiotic-resistant microorganisms [26, 27].

Nowadays, numerous studies have been addressed in the development of bio-derived TiO_2_-polymeric nanocomposites for diverse applications [28, 29]. However, limited scientific reports are available on the antibacterial and anticancer potential of TiO_2_-reinforced biopolymers [30–32]. The photocatalytic effect of biodegradable aliphatic polyester films incorporated with TiO_2_ particles was screened for their competence for the removal of volatile organic components [33]. A study conducted by Tang described the preparation of polycaprolactone-TiO_2_ nanocomposites by a solution-casting method and evaluated their mechanical and self-cleaning properties [34]. A biopolymer prepared from waste cooking oil doped with TiO_2_ fillers was reported as a surface coating for indoor and outdoor building applications [35]. Nevertheless, the aforementioned studies have not been screened for the antimicrobial effects of the film. Few reports are available in the literature with regard to the synthesis of TiO_2_ coated oil-based polymeric nanoparticles that were evaluated for antibacterial activity. Recently, TiO_2_ nanoparticles loaded polyethylene films have shown a potential antimicrobial effect against *Staphylococcus aureus*, suggesting that PE/TiO_2_ composite film might prevent the high relative humidity throughout the packing system, delaying spoilage of food and thus increasing their shelf life. Hence, these films can serve as the best candidate for the food packaging system [36]. Another study conducted by Feng et al. revealed that PLA/TiO_2_ nanofibers and films prepared by electrospinning and solution casting methods exhibited strong antibacterial effects against *Escherichia coli* and *S. aureus*. The results of this study concluded that both the nanocomposite membranes satisfied the requirements of food packaging materials [37].

The present study reports the synthesis and characterization of *P. cylindraceus* oil/TiO_2_/polyethylene glycol polymeric bionanocomposite comprised *P. cylindraceus* oil and polyethylene glycol decorated with anatase TiO_2_ nanoparticles. The synthesized bionanocomposite was evaluated for antibacterial and anticancer activities against various pathogenic strains and cancer cell lines.

## 2. Materials and Methods

### 2.1. Instrumentation

All spectrophotometric measurements and the characterization of the synthesized nanoparticles were carried out by measuring the UV-Vis spectrum of the as-prepared TiO_2_ nanoparticles using an Ultrospec 2100-Biochrom spectrophotometer (Biochrom Ltd., Cambium, Cambridge, UK). Fourier-transform infrared (FTIR) spectra of the formed nanoparticles and their bionanocomposites were recorded using PerkinElmer FT-IR spectrophotometer (PerkinElmer Ltd., Yokohama, Japan). The morphologies of TiO_2_ NPs and the polymeric *P. cylindraceus* oil*/*TiO_2_*/*PEG bionanocomposite were measured by scanning electron microscope (JEM-2100F, JEOL Ltd., Akishima, Tokyo, Japan) and JEM-1400 transmission electron microscope (JEOL Ltd., Akishima, Tokyo, Japan). XRD patterns of TiO_2_ nanoparticles and the bionanocomposite were obtained by Siemens D-5000 diffractometer (Siemens, Erfurt, Germany). The pH-meter Metrohm model 744 (Metrohm Co., Herisau, Switzerland) was used to control the pH condition of the test solution. Distilled water (H_2_O) was used throughout the experimental study. Thermal stability analysis was conducted using a Shimadzu thermogravimetric analyzer (TGA-502 model). Nikon ECLIPSE fluorescence microscopy (Ti-E, Japan) was used to analyze cancer cell apoptosis.

### 2.2. Chemicals and Reagents

Titanium (IV) nitrate tetrahydrate (Ti(NO_3_)_4_.H_2_O, ≥99.9%), pure grade of polyethylene glycol (PEG), analytical-grade acetone (anhydrous, ≥99.0%), ethanol (96%), 3% of glutaraldehyde in phosphate, 3-(4,5-dimethylthiazol-2-yl)-2,5-diphenyltetrazolium bromide (MTT), lactate dehydrogenase (LDH) rhodamine 123 dye, acridine orange/ethidium bromide (AO/EtBr) dye, dichloro dihydro fluorescein diacetate (DCFH-DA), and anhydrous sodium sulfate were acquired from Sigma-Aldrich **(**Hamburg, Germany). Ciprofloxacin (5 *μ*g/disc, MASTDISCS™, Mast Diagnostics Ltd.), vancomycin (Glaxo SmithKline Pharmaceuticals Ltd.), and gentamycin (Alpha Laboratories Ltd.) were purchased from local drug stores.

### 2.3. Botanical Material

*Plectranthus montanus* Benth. (syn. *Plectranthus cylindraceus* Hoechst. Ex. Benth.) was collected from the Abha region of Saudi Arabia in March 2018. Dr. Mohamed Yousef, a taxonomist at the Pharmacognosy Department of the King Saud University, identified the plant material, and a voucher specimen (P-5-2018) was deposited in the same department. Aerial parts of the collected plant were sun-dried to remove the moisture content. The dried plant material was coarse powder in a mixer grinder for oil extraction. The botanical sample was kept at 4°C in the refrigerator until further use.

### 2.4. Bacterial Strains and Cancer Cell Line

Four bacterial strains: *S. aureus* (ATCC 25923), *E. coli* (ATCC 25922), *Pseudomonas aeruginosa* (ATCC 25566), and *Salmonella typhi* (ATCC 27736) and human lung carcinoma cells were used to test the antibacterial and anticancer effect of *P. cylindraceus* oil and *P. cylindraceus* oil/TiO_2_/PEG bionanocomposite. Bacterial strains and cancer cell lines were supplied by the Microbiology Department of the King Khalid Hospital, Riyadh, Saudi Arabia, and Research Center of King Faisal Hospital, Riyadh, Saudi Arabia, respectively.

### 2.5. Extraction of *P. cylindraceus* Oil

Powdered aerial parts (300 g) of *P. cylindraceus* were subjected to hydrodistillation in a Clevenger apparatus for 4 h to yield colorless oil by obeying the previous method of Khan et al. with slight modification [38]. The obtained volatile oil was dried over anhydrous sodium sulfate as a dehydrating agent and stored in the refrigerator at 4°C for subsequent use. The yield of the volatile oil obtained from the *P. cylindraceus* was 1.2% on the basis of fresh weight.

### 2.6. Gas Chromatography-Mass Spectrometry (GC-MS) Analysis of Essential Oil

The qualitative and quantitative of volatile oil was carried out on Hewlett-Packard-5890 series II plus gas chromatograph coupled with HP-5989 mass spectrometer. The separation was performed in HP5-MS capillary column (25 m × 0.25 mm) coated with 0.50 *µ*m 5% phenyl in 95% methylpolysiloxane, programmed at 70–250°C temperature with a flow rate of 3°C/min. Helium was used as a carrier gas at 1.9 mL/min at a steady flow rate. The 250°C and 280°C temperatures were adjusted for the injector and interface, respectively. Electron ionization mass spectra of the components were obtained at temperature 250°C and ionization voltage 70 eV. Finally, the obtained unknown compounds were identified by comparing spectra available from the Wiley 8 and NISTO 5 database mass spectral library. AMDIS32 software was used to calculate the retention indices (IR) values and Linear retention indices obtained for the compounds were compared with those published in the literature [39]. The constituents of *P. cylindraceus* oil were identified on the basis of retention time, comparison with Wiley, 2008 database library, and fragmentation pattern of components with those already reported in the literature [40].

### 2.7. Preparation of TiO_2_ Nanoparticles

The collected aerial parts of *P. cylindraceus* (25 g) were washed thoroughly with water and boiled in 200 mL of distilled water at 80°C for 20 min. The obtained extract was filtered using nylon mesh (spectrum) followed by a millipore hydrophilic filter (0.22 *µ*m). The resulted aqueous extract was used to prepare TiO_2_ nanoparticles. Briefly, 20 mL of prepared *P. cylindraceus* extract was added to 80 mL of titanium (IV) nitrate tetrahydrate (1.0 × 10^−3^ mol L^−1^) with continuous stirring for 24 h at room temperature until the formation light green precipitate of TiO_2_ NPs. The resulted nanoparticles were centrifuged, filtered, and dried in an air oven (Scheme 1(a)).

### 2.8. Preparation of the Polymeric *P. cylindraceus* Oil/TiO_2_/PEG Bionanocomposite

The fabrication of an ultrafine plain film of PEG polymer and *P. cylindraceus* oil was performed by mixing 10% of PEG dissolved in 5 mL acetone with 5–15% of *P. cylindraceus* oil under magnetic stirring for 12 h at ambient temperature until the formation of the homogeneous composite. The obtained plain *P. cylindraceus* oil/PEG composite was decorated with TiO_2_ NPs by mixing 5 w% of *P. cylindraceus* oil and 5 w% TiO_2_ NPs suspended in the polymeric mixture and subjected to vigorous shaking for 6 h at room temperature. The polymeric *P. cylindraceus* oil/TiO_2_/PEG bionanocomposite film was obtained and kept aside for further investigation (Scheme 1(b)).

### 2.9. Characterization of TiO_2_ Nanoparticles and *P. cylindraceus* Oil/TiO_2_/PEG Bionanocomposite

Various spectroscopic analyses, including ultraviolet-visible (UV-vis.), Fourier-transform infrared (FTIR), and X-ray diffraction (XRD), were carried out to characterize the TiO_2_ nanoparticles and their polymeric bionanocomposites. The nanoparticles and polymeric bionanocomposites were further confirmed by microscopic analysis using a scanning electron microscope (SEM) equipped with energy dispersive X-ray (EDX) and transmission electron microscopy (TEM).

### 2.10. Thermal Stability and Hydrolytic Degradation of the Bionanocomposite

The thermal stability of the prepared bionanocomposite film was investigated by using thermogravimetric analysis (TGA, Seiko Exstar 6300, Tokyo, Japan). Around 5 mg of sample was heated from a temperature range of 10 to 600°C at a 10°C/min heating rate under a constant flow of argon of a Shimadzu thermogravimetric analyzer (TGA-502 model).

The hydrolytic degradation analysis of bionanocomposite film was investigated by controlling the pH and temperature of the system according to ASTM F1635-11 [41]. The analysis was performed for 8 weeks. Saline phosphate buffer (pH 7.4) was used to test the hydrolytic degradation of bionanocomposite in triplicates. The binaocomposite film was kept in 10 mL PBS solution and heated in a water bath at 37°C. The film was removed at different time intervals (2^nd^, 4^th^, 6^th^, and 8^th^ weeks) from the controlled medium and oven-dried at 60°C. Subsequently, the weight loss of the bionanocomposite film was monitored through gravimetric analysis together with the degradation test. Time zero was adjusted as before initiating the experiment, and the measurements were recorded at the time of withdrawals of the film. No results of weight loss were obtained at 8^th^ withdrawal due to the high deterioration of the bionanocomposite film. The results of weight loss were obtained through the following equation:

(1) $$\begin{array}{c} M=M_{0}-M_{f}, \end{array}$$

where *M*, *M*_0_, and *M*_*f*_ are the weight loss, mass of the film before degradation, and mass of the film at different removal times, respectively.

### 2.11. Antibacterial Effect of *P. cylindraceus* Oil and Bionanocomposite

The antibacterial activity of the oil and as-prepared bionanocomposite was evaluated by the disc diffusion method [42]. To culture the microorganisms, Mueller–Hinton agar plates were incubated at 37°C for 18 h. A bacterial cell density of 10 × 10^8^ UFC/mL was adjusted with a sterile saline solution. To obtain the uniform bacterial growth, a sterile swab was dipped in each microbial suspension and used to spread microorganisms over the test and control plates. Different concentration (25–100 *µ*gmL^−1^) of 10 *µ*L of each *P. cylindraceus* oil and *P. cylindraceus* oil/TiO_2_/PEG bionanocomposite was loaded on the surface of the sterile disc. Afterwards, the plates were incubated for 24 h at 37°C, and the zones of inhibition were determined in millimeters. Ciprofloxacin (5 *μ*g/disc) containing disc was used as a reference control for bacterial inhibition. All the experiments were performed in triplicates, and the mean inhibition diameter was calculated. The activity was evaluated as either sensitive or resistant with a cutoff value equal to 10 mm.

### 2.12. Determination of Bacteriostatic and Bactericidal Concentrations

Minimum inhibitory concentrations (MIC) of *P. cylindraceus* oil/TiO_2_/PEG bionanocomposite against methicillin-resistant *S. aureus* and *E. coli* were determined by the microdilution method using Mueller–Hinton broth. Vancomycin and gentamycin were used as a positive reference control for *S. aureus* and *E. coli* strains, respectively. Minimum bactericidal concentration (MBC) of polymeric bionanocomposite was expressed as spreading aliquots of tubes with no visible growth and the first turbid tube in the MIC series. A sterile rod was used to spread uniformly the aliquots of treated samples on nutrient agar plates and incubated at 37°C for 12 h.

### 2.13. Morphological Study of *S. aureus* and *E. coli* (SEM)

The morphological changes in treated and untreated *S. aureus* and *E. coli* by the prepared *P. cylindraceus* oil/TiO_2_/PEG bionanocomposite were studied under scanning electron microscopy. The treated microorganisms were cut into 5–10 mM pieces and fixed on a glass slide for 1 h in 3% of glutaraldehyde in phosphate buffer saline solution. The treated tissues were dehydrated with ethanol and dried with carbon dioxide. Silver pain vacuum coated with gold-palladium alloy was used to mount the dry tissues on the aluminum stubs and examined under SEM with 15 kV acceleration voltage.

### 2.14. Anticancer Effect of *P. cylindraceus* Oil and Bionanocomposite

The cytotoxic effect of *P. cylindraceus* oil and polymeric bionanocomposite against human lung carcinoma (A549) cell lines was performed according to the previously reported method [43]. The A549 cancer cells were kept in a DMEM medium comprised 10% FBS, 100 mg mL^−1^ streptomycin, 2 mM glutamine, and 100 IU mL^−1^. The cell cultures were maintained in a humidified incubator at 37°C with a continuous flow of 5% CO_2_. A 1 × 10^4^ cells/well concentration of A549 cell culture was separately seeded in 96 well plates. The cells were treated with different concentrations of *P. cylindraceus* oil and polymeric bionanocomposite (0 to 200 *µ*g mL^−1^) and incubated for one complete day. After 24 h of incubation, 100 *µ*L of MTT (3-(4,5-dimethylthiazol-2-yl)-2,5-diphenyltetrazolium bromide) was added to treated cells and further incubated for 4 h at 37°C. After 4 h incubation, a purple-colored formazan dissolved in 100 *µ*L of dimethyl sulfoxide was then added. After 30 min, optical density was recorded on ELISA multiwell plate reader at 570 nm for calculating IC_50_ values. A lactate dehydrogenase (LDH) leakage assay was performed to assess the damage of the cell membrane and loss of membrane integrity. Rhodamine 123 staining was employed to analyze the changes that occurred in mitochondrial membrane potential (ΔΨm) after the treatment of bionanocomposite. All the experiments were performed in triplicates to avoid errors.

### 2.15. Acridine Orange/Ethidium Bromide (AO/EtBr) Staining

The ability of *P. cylindraceus* oil *and P. cylindraceus* oil/TiO_2_/PEG bionanocomposite to induce apoptosis (A549 cells) was evaluated using double staining acridine orange/ethidium bromide (AO/EtBr). The staining procedure was performed according to the previously reported method [44]. Two six-well plates were individually seeded with A549 cancer with respect to IC_50_ concentrations of *P. cylindraceus* oil and polymeric bionanocomposite and were incubated for one day. Acridine orange (100 *μ*g mL^−1^) and ethidium bromide (100 *μ*g mL^−1^) fluorescent dyes were mixed with respective cells and incubated in the dark for 30 min at 37°C. Cells were immediately viewed under a fluorescence microscope with 500 nm excitation wavelength, and the emission was recorded at 570 nm. The AO/EtBr double staining test mechanism revealed that cells having normal nuclear chromatin represent green nuclear staining confirmed that AO is picked up only by viable cells. However, apoptotic cells containing condensed chromatin portray orange to red nuclei revealed that EtBr was picked up by nonviable cells.

### 2.16. Dichloro Dihydro Fluorescein Diacetate (DCFH-DA) Assay

The DCFH-DA staining was applied to estimate the intracellular ROS generation in A549 cancer cells by *P. cylindraceus* oil and *P. cylindraceus* oil/TiO_2_/PEG bionanocomposite. Two six-well plates were individually seeded with A549 cancer cells and treated separately with *P. cylindraceus* oil and polymeric bionanocomposite. The treated cells were incubated for 24 h, rinsed with 1x cold phosphate buffer saline (PBS, pH 7.4), stained with 10 *μ*g/10 *μ*L DCFH-DA and kept in dark for 39 min. The level of ROS generation was evaluated under the fluorescence microscope. The above assay was performed according to the previously reported procedure and in triplicates [45].

### 2.17. Photocatalytic Effect of the Bionanocomposite

The photocatalytic effect of polymeric bionanocomposite was estimated on the basis of its ability to degrade the methylene blue (MB) dye under visible and UV radiations. The ultraviolet source used for the experiment was a Mercury vapor lamp with 120 W. A methylene blue stock solution (20 *µ*g mL^−1^) was prepared. Ten milliliter of polymeric bionanocomposite was mixed with 100 mL of dye solution under continuous magnetic stirring for 1 h in the dark to enhance the equilibrium balance between MB and photocatalyst prior to exposure to sunlight and UV irradiations. The reaction mixture was irradiated by the light source, and after each 30 min time interval, around 2 mL of the suspension was taken up and centrifuged to remove the suspended nanoparticle. UV-visible spectrophotometer was employed to determine the rate of dye degradation at 660 nm, and the degradation percentage was calculated by applying the following formula:

(2) $$\begin{array}{c} \%\text{ of degradation }=\;\frac{C_{i}-C_{f}}{C_{i}}\times 100, \end{array}$$

where *C*_*i*_ and *C*_*f*_ were the initial and final concentrations of dye at a time interval “*t*,” respectively.

## 3. Results and Discussion

### 3.1. Chemical Composition of *P. cylindraceus* Oil by GC-MS

Hydrodistillation of fresh aerial parts of *P. cylindraceus* resulted in the extraction of a pleasant smelling colorless essential oil with an excellent yield of 0.42% (v/w). Qualitative and quantitative GC-MS analysis of *P. cylindraceus* oil identified 30 constituents that accounted for 96.54% of total oil composition. The identified compounds with their linear indices (LRI) and relative content are summarized in Table 1. The essential oil is composed of about 90% of monoterpenes of which 70% were oxygenated monoterpenes while 20% were nonoxygenated monoterpene. Seven of the detected constituents present in the oil were oxygenated sesquiterpenes. Camphor (38.85%) and 1,8-cineol (21.84%) were present as the major compounds of *P. cylindraceus* oil. Other classes of constituents such as oxygenated aliphatic alkanes (1.4%), diterpenes (1.2%), and aromatic and aliphatic hydrocarbons (0.4) were found in minute quantities (Figure 1).

### 3.2. Characterization of TiO_2_ Nanoparticles and Bionanocomposite

Different spectroscopic and microscopic investigations were employed to characterize the formation of TiO_2_ nanoparticles and their bionanocomposites. The UV-Vis screening of TiO_2_ nanoparticles (from 250 to 500 nm) prepared by *P. cylindraceus* aqueous extract showed an absorption peak at a wavelength of 350 nm (Figure 2(a)). The obtained result was in agreement with the previously reported synthesis of TiO_2_ nanoparticles [46]. A particle size analyzer was used to calculate the average particle size of the formed TiO_2_ nanoparticles, and the mean average value was found to be around 60 nm (Figure 2(b)). The size and shape of TiO_2_ nanoparticles were viewed under SEM, and images were picked at different magnifications (30,000x and 50,000x) showed irregular shape nanoparticles with particle size ranging from 68 to 88 nm (Figures 3(a) and 3(b)).

Gradual addition of *P. cylindraceus* oil (5–15%) was applied to select the suitable oil concentration to fabricate the suggested *P. cylindraceus* oil/TiO_2_/PEG bionanocomposite. Around 5% of *P. cylindraceus* oil was initially added, but this quantity of oil could not give a well-characterized bionanocomposite. Therefore, gradual increments of *P. cylindraceus* oil were continued up to 15 w%. It was observed that 15w% of *P. cylindraceus* oil provides well-characterized polymeric *P. cylindraceus* oil/PEG solution. The surface morphology of PEG, the prepared plain polymeric mixture, and the synthesized *P. cylindraceus* oil/TiO_2_/PEG bionanocomposite was examined under SEM using 30,000x magnifications. The surface morphology of 100 nm of PEG at 30,000x showed a smooth and uniform polymeric matrix distribution (Figure 4(a)). The SEM images of plain *P. cylindraceus* oil at 30,000x magnifications showed the irregular coagulant mass with rounded oil droplets and tiny pores (Figures 4(b) and 4(c)). Furthermore, the SEM images of the synthesized bionanocomposite at the same magnification indicated the irregular structure of TiO_2_ nanoparticles with particle sizes ranging between 68 and 88 nm (Figure 4(d)).

The XRD pattern of TiO_2_ nanoparticles synthesized from aqueous *P. cylindraceus* extract was studied. The obtained results revealed that the structure was irregular. These results were in good agreement with JCPDS card number 21–1272. The XRD peaks were observed at 26°, 37°, 46°, 51°, 56°, 63°, and 74° corresponding to miller index values (1 0 1), (0 0 4), (2 0 0), (1 0 5), (2 1 1), (2 0 4), and (2 1 5), respectively (Figure 5(a)). It was noticed that as the width of the peak increases, there is a decrease in particle size, indicating that the formed particles were in nanoscale. To confirm the dispersion of *P. cylindraceus* oil and TiO_2_ nanoparticles in the polymeric matrix PEG, XRD analysis with Cu k*α* radiation (*λ* = 1 540 Ǻ) over Bragg angles in a range from 10 to 80 degrees, current-voltage 50 mA, and 35 kV was applied. The outcomes of XRD analysis demonstrated that no significant peak was recorded for the polymeric solution of PEG (Figure 5(b)-A); this was due to the amorphous nature of the plain polymer [47]. However, the XRD pattern of *P. cylindraceus* oil-PEG showed a broad peak near ∼20 degrees (Figure 5(b)-B), this could be due to the dispersion of *P. cylindraceus* oil in the PEG matrix causing a remarkable change in the peak intensity. However, the XRD spectrum of the synthesized *P. cylindraceus* oil/TiO_2_/PEG bionanocomposite showed the appearance of distinct peaks at 39.26°, 42.15°, 56.83°, and 73.52° revealed that Bragg's reflection was from TiO_2_ (101), TiO_2_ (004), TiO_2_ (200), and TiO_2_ (215) (Figure 5(b)-C). The observed peaks clearly confirmed the decoration of TiO_2_ nanoparticles over the surface of the plain polymeric-oil mixture, resulting in the formation of bionanocomposite film.

EDX analysis of PEG and the bionanocomposite was investigated using an EDX equipped with SEM. Figures 6(a) and 6(b) show the surface morphology of the plain polymer and the synthesized bionanocomposite. The presence of TiO_2_ nanoparticles indicated that the metal oxide was dispersed well in the polymeric matrix. Two signals representing C and O for PEG were displayed. However, the synthesized bionanocomposite showed the presence of distinct signals for C, O, and Ti (Figures 6(c) and 6(d)). No other elemental impurity was observed. The EDX results confirmed that the bionanocomposite was successfully fabricated and well distribution of *P. cylindraceus* oil and TiO_2_ nanoparticles in the polymeric matrix PEG.

### 3.3. Thermal Stability and Hydrolytic Degradation of the Bionanocomposite

The thermal stability of bionanocomposite has a great influence on inherent properties and strong intermolecular interaction between the bionanocomposite molecules. An increase in thermal energy as compared to bond dissociation energy greatly affects the dissociation of the polymeric chain of bionanocomposite [48]. The interaction between the surfaces of organic and inorganic nanomaterials was confirmed by thermogravimetric analysis. The stability of bionanocomposite was evaluated at different weight percent (5 w%, 10 w%, and 15 w%) of PEG/TiO_2_ NPs (Figure 7). The results showed that weight reduction started at 130°C, and measured values were 150, 175, and 230°C for the aforementioned bionanocomposite film. It was noticed that around 10% of water was lost from the surface of the bionanocomposite film between 175 and 230°C, suggesting that 230°C is the maximum thermal stability limit. Therefore, the outcomes revealed that an increase in the PEG weight percent resulted in an increase in carbonaceous material residual weight generated by polymer decomposition. However, the hydrolytic degradation showed different trends in the behavior of weight loss in the bionanocomposite. The results revealed that there was no loss of bionanocomposite weight at the beginning of the experiment. However, 5.70% and 13.54% of its weight was lost in the 2^nd^ and 6^th^ week, respectively (Table 2). It may be hypothesized that the degradation was affected by the addition of TiO_2_ NPs and PEG, which triggered the water penetration into the system that resulted in the diminution of polymeric chain and enhanced the disintegration of the system.

### 3.4. Antibacterial Effect of the Bionanocomposite

The antibacterial efficacy of the pure *P. cylindraceus* oil and *P. cylindraceus* oil/TiO_2_/PEG bionanocomposite were determined against microbes based on the zone of inhibition. *P. cylindraceus* oil and polymeric bionanocomposite were subjected to antibacterial tests against four bacterial species, namely *S. aureus*, *E. coli*, *P. aeruginosa*, and *S. typhi*. Preliminary screening results revealed that the as-synthesized polymeric bionanocomposite showed much greater antibacterial potential compared to pure *P. cylindraceus* oil at similar proportions. At the highest sample concentration (50 *µ*gmL^−1^), polymeric bionanocomposite displayed a nearly twofold greater bactericidal effect compared to *P. cylindraceus* oil as measured using the disc diffusion test. After 48 h incubation, the zones of inhibition of bionanocomposite and *P. cylindraceus oil against S. aureus and E. coli* were (20.03 + 1.20 and 25.50 ± 1.08 mm) and (14.52 + 0.68 and 16.12 ± 0.56 mm), respectively. As shown in Table 3, *P. cylindraceus* oil and polymeric bionanocomposite exhibited the strongest antibacterial effect towards *E. coli* and *S. aureus* (Figure 8(a)). *P. cylindraceus* oil has been reported to provide the benefits of antimicrobial activity and medicinal value [49]. *P. cylindraceus* oil is dominated by monoterpenes; especially camphor and 1,8-cineol have extensive antibacterial potential because Gram-positive and Gram-negative bacteria were found susceptible to these oils [50, 51]. The strong bactericidal effect of polymeric bionanocomposite may be attributed to TiO_2_ nanoparticles that strongly bond with electron-donating groups in bioactive compounds containing oxygen, sulfur, and nitrogen. These nanoparticles disturb the cell boundary of microorganisms and as a result, the outermost rigid cell layer lost its protection. The small size of TiO_2_ nanoparticles facilitates the easy penetration to cell membranes, and monoterpenes present in oil disturb the lipid fraction of the plasma membrane of bacteria, resulting in alterations of membrane permeability and leakage of intercellular content. Also, the TiO_2_ nanoparticles and their ions have the ability to produce free radicals (reactive oxygen species, hydroxyl ion, superoxide ion, singlet oxygen, and hydrogen peroxide) that induces oxidative stress [52]. The ROS can permanently destroy the microbes and result in the death of microbes. There are two probable mechanisms involved in antibacterial action of as-synthesized polymeric bionanocomposite, that is, photogeneration of free radicals or by the intracellular interaction between microbial cell membrane and nanoparticles (negative charge of the outermost layer of cell membrane with positive charge of TiO_2_ ions) resulting in microbial growth inhibition and inducing the demise of microbes. A steady S-metal group is formed when the ions released from TiO_2_ nanoparticles bond with thiol or sulfhydryl groups (–SH) and proteins of the cell membrane with the loss of hydrogen ion, reducing the cell permeability and resulted in the death of the cell [53]. However, ROS generation contributes to the disruption of DNA, enzymes, proteins, and lipids. The enzyme inhibition caused by polymeric bionanocomposite was found to be the most efficient mechanism as it destroys the assimilatory food pathway and induces cell death [54]. The mechanism of polymeric bionanocomposite can proceed via two kinetic processes utilizing their ability to penetrate the bacterial cell membrane and killing the microorganism or by phagocytosis of TiO_2_ nanoparticles by the mononuclear phagocyte system (Scheme 2). Antibacterial potentials of *P. cylindraceus* oil and polymeric bionanocomposite against *S. aureus* and *E. coli* are demonstrated in Scheme 2. Also, antibacterial results showed that polymeric bionanocomposite as well as pure oil were more susceptible against *E. coli* (Gram-negative) bacteria as compared to *S. aureus* (Gram-positive) due to differences in cell wall composition. The cell wall of *E. coli* contains a thin peptidoglycan layer in contrast to *S. aureus* [55]. Thus, the result obtained confirmed that polymeric bionanocomposite exerted a remarkable bactericidal effect than pristine *P. cylindraceus* oil. The zone of inhibition against *P. cylindraceus* oil and polymeric bionanocomposite against *S. aureus* and *E. coli* is shown in Figure 8(a).

### 3.5. MIC and MBC of the Polymeric Bionanocomposite against *S. aureus* and *E. coli*

Agar well diffusion procedure was applied to determine the bacteriostatic and bactericidal concentrations of *P. cylindraceus* oil/TiO_2_/PEG bionanocomposite. The lowest concentration required for inhibition of visible growth of *S. aureus* and *E. coli* was assessed after 24 h at 37°C. The gradual increase in polymeric bionanocomposite concentration (5–1,280 *μ*g mL^−1^) has shown a significant reduction in bacterial cell viability (*p* < 0.05). The 320 *μ*g mL^−1^ represents the MIC for the *S. aureus* and *E. coli* as depicted in Figure 8(b) (A and B). MBC for *S. aureus* and *E. coli* was displayed at 640 and 1,280 *μ*g mL^−1^, respectively, for the polymeric bionanocomposite (Table 4). The antibacterial properties of polymeric bionanocomposite were enhanced in contrast to pristine *P. cylindraceus* oil, due to the small size of TiO_2_ nanoparticles that provide a more dominant attack to the cell membrane of the microorganisms [56].

### 3.6. Morphological Study of *S. aureus* and *E. coli*

The effect of polymeric bionanocomposite on the surface morphology of *S. aureus* and *E. coli* was inspected under SEM. The treatment of polymeric bionanocomposite has changed the shape and size of selected microbes due to the coating of TiO_2_ nanoparticles on the surface of microbial cells as illustrated in Figures 9(b) and 9(e). The polymeric bionanocomposite can easily penetrate the peptidoglycan layer of the cell membrane of *S. aureus* and *E. coli*, leading to the destruction of the cell membrane, leakage of cell ingredients, and consequently resulting in the death of the microbial cell (Figures 9(c) and 9(f)) [52]. The untreated microbial cells were selected as a positive control for the comparison (Figures 9(a) and 9(d)).

### 3.7. Anticancer Effect of the Polymeric Bionanocomposite

Lung cancer is among the most widespread form of carcinoma experience in humans and the leading cause of cancer-related death worldwide. Epidemiological studies have shown that among all types of cancer, 17.6% of total cancer deaths occur due to lung cancer [57]. Nonsmall lung cancer (NSCLC) is the main sponsor of total lung cancer, which is classified further into large cell carcinoma (2.9%), squamous cell carcinoma (20%), and adenocarcinoma (35%) [58]. Adenocarcinomic human alveolar basal epithelial cells (A549) are frequently used as *in vitro* model systems for the investigation of NSCLC. The major responsible determinants of lung cancer are environmental and lifestyle factors including air pollution, smoking, alcohol, lack of physical activity, occupational exposure, and diet [59]. The sudden rise in lung cancer mortality rate is due to the lack of efficient diagnostics and therapeutic strategies. The treatment used for lung cancer includes surgery, chemotherapy, and radiotherapy alone or in combination depending on the stage of cancer. Gemcitabine in combination with cisplatin is FDA-approved chemotherapeutic drug that has been utilized as a primary drug for lung cancer therapy. Recently, combinatorial drug therapy has gained much attention due to the improvement of the therapeutic efficacy of the drug. Cisplatin in combination with paclitaxel, gemcitabine, and docetaxel drugs have expressed enhanced therapeutic efficiency [60, 61]. However, the majority of these chemotherapeutic drugs are very expensive and associated with adverse side effects such as neuronal damage, skin irritation, and acute pain. Hence, there is a serious demand for the development of nontoxic, cost-effective, ecofriendly, and targeted drugs for cancer treatment. Nanoparticles possessing unique physiochemical features offer an extraordinary interaction with proteins, nucleic acids, and lipids present on the surface of cells and within the cell body, which might establish new routes for the diagnosis and treatment of cancer [62]. Recently, several bio-based polymeric nanocomposites have shown outstanding anticancer properties against various types of cancer [63]. In the present study, the anticancer effect of *P. cylindraceus* oil/TiO_2_/PEG bionanocomposite prepared through a biogenic route using *P. cylindraceus* oil was evaluated against lung cancer cells (A549).

### 3.8. Antiproliferative Effect of the Polymeric Bionanocomposite

MTT assay and LDH leakage assay were applied to assess the *in vitro* cytotoxic activity of *P. cylindraceus* oil/TiO_2_/PEG bionanocomposite.  Figure 10(a) clearly depicts that polymeric bionanocomposite exhibited potent cytotoxic activity against A549 cancer cell lines in a dose-dependent manner with 42.7 ± 0.25 *μ*g mL^−1^ IC_50_ value, in contrast to cisplatin positive control (IC_50_ value of 27.6 ± 0.018 *μ*g mL^−1^). Morphological changes occurred in the cell and membrane damage was analyzed under phase-contrast microscope. Results revealed a high-density cell population with normal epithelial morphology in the control group, whereas rounded and shrunk cells, condensed chromatin, formation of apoptotic body, and protrusions of membrane were noticed in the cells treated with polymeric bionanocomposite and positive control (Figure 10(b)). The activation caspase cascade caused by polymeric bionanocomposite and positive control might be responsible for morphological changes, wherein the component poly (ADP-ribose) polymerase (PARP) needed for the repair of DNA would be cleaved [64]. Cellular uptake of nanoparticles by endocytosis or macropinocytosis would initiate the ROS generation, trigger the apoptotic pathway, and eventually lead to cell demise [65].

The cellular or tissue damage was assessed on the basis of the level of lactate dehydrogenase (LDH) in the extracellular medium. LDH is a cytoplasmic soluble enzyme, released during the disruption of the cell membrane into the extracellular matrix. Thus, the increased level of LDH indicates cellular toxicity [66]. The cytotoxic potential of polymeric bionanocomposite was further validated by the LDH leakage assay. The results showed that the increase in the percentage of LDH leakage was found concentration-dependent in polymeric bionanocomposite-treated cells (Figure 10(c)). The above results were in accordance with the previous reports that TiO_2_ nanoparticles treatment would permeabilize the cell membrane, allowing the LDH leakage in lung cancer cells, causing cell demise [67].

### 3.9. Bionanocomposite-Induced Apoptosis via ROS-Mediated DNA Damage

Chemotherapeutic drugs and radiation therapy induce the death of cancer cells by the activation of the ROS-mediated apoptosis pathway. An increase in the levels of ROS leads to various pathological incidences such as inflammation, lipid peroxidation, protein oxidation, and DNA damage. ROS generation is considered to participate in several cellular events including inflammation, DNA damage, senescence mutation, and apoptosis [68]. In the current study, the levels of intracellular ROS were measured in A549 cancer cells to determine the mechanism behind the anticancer properties of polymeric bionanocomposite. Spectrofluorometric results showed that the fluorescence intensity in polymeric bionanocomposite treated groups was increased twofold in comparison to the control group (Figure 11(c)). The fluorescent microscopic analysis was applied to validate the results, which exhibited an enhanced fluorescent green intensity in the polymeric bionanocomposite treated cells, in contrast to the positive control and control, indicating a rise in ROS level (Figure 11(d)). These results confirmed that apoptosis induced by polymeric bionanocomposite was associated with the accumulation of ROS in A549 cancer cells.

### 3.10. Estimation of Loss of Mitochondrial Membrane Potential

One of the key players required for activation of apoptotic pathway is the loss of mitochondrial membrane potential (MMP Ψm) [69]. The disturbance of MMP in A549 cancer cells in polymeric bionanocomposite treated cells was examined by using Rhodamine 123 dye. In contrast to control cells, a potent reduction (*p* < 0.05) in fluorescence intensity nearly threefold was noticed in polymeric bionanocomposite treated cells, representing MMP disruption (Figure 11(b)). A reduction in fluorescent intensity was observed in the polymeric bionanocomposite treated cell under a fluorescence microscope, validating the spectrofluorometric results and further confirming the fact that polymeric bionanocomposite would cause a potential loss in MMP (Figure 11(a)).

### 3.11. Polymeric Bionanocomposite-Induced Apoptosis in A549 Cells

The predominant mechanism of action of chemotherapeutics used in cancer treatment proceeds by triggering the apoptotic pathway to destroy the cancer cells [70, 71]. AO/EtBr dual staining procedure was applied to determine the rate of apoptosis persuade by polymeric bionanocomposite.  Figure 12(a) displays the presence of uniform green-colored cells in the control vehicle, representing the presence of live cells (early apoptotic cells) in the range of 500 to 530 nm under a fluorescent microscope. However, polymeric bionanocomposite treated cells displayed the presence of red- and orange-colored cells, representing dead cells (late apoptotic cells) in the range of 510 to 595 nm under a fluorescent microscope, while in cisplatin-treated cells, dual stained green and orange-colored cells were found, indicating the necrosis. The results of the quantitative analysis showed that a significant increase in apoptotic cells was observed in polymeric bionanocomposite-treated cells (80.3 ± 0.01% dead and 19.7 ± 0.02% live cells) while compared to nontreated (88.9 ± 1.20% live and 11.02 ± 0.86% dead cells). Cisplatin-treated cells (positive control) showed the presence of 36.2 ± 0.08% live cells and 63.7 ± 0.05% apoptotic cells (Figure 12(b)). The results demonstrated that the polymeric bionanocomposite led to the apoptotic cell demise of A549 cancer cells.

To get further understanding of the mode of cell demise stimulated by polymeric bionanocomposite, 4′,6-diamidino-2-phenylindole (DAPI) staining was performed. As shown in Figure 12(c), the polymeric bionanocomposite treatment caused condensation of chromatin and morphological alteration in the nucleus of A549 cancer cells, illustrating the fact that the apoptotic potential of polymeric bionanocomposite is completely dependent on the production of ROS levels, which in turn has resulted in oxidative stress-mediated cell death in A549 cancer cells. The results concluded that TiO_2_ nanoparticle present on the surface of the bionanocomposite film of polymeric bionanocomposite enhanced the production of intracellular ROS level, creating oxidative stress, disrupting MMP, consequently activating apoptotic intrinsic pathway and ultimately causing the death of the cell. Above all, ROS, MTT, LDH, AO/EtBr, and DAPI results confirmed an enhanced anticancer potential against A549 cell lines using *P. cylindraceus* oil/TiO_2_/PEG bionanocomposite compared to that of the previous similar report [72].

### 3.12. Safety Determination of the Bionanocomposite in PBMC

*In vitro* toxicity studies were conducted as an alternate method to validate the toxicological profile of the newly identified drug [73]. For the determination of immunotoxicity and dosage limit of the new drug constituent under investigation, human peripheral mononuclear cells (PBMC) were applied *in vitro* model [74]. MTT assay was used to determine the *in vitro* cytotoxic potential of polymeric bionanocomposite in PBMC.  Figure 12(d) demonstrates that the prepared bionanocomposite treatment induced no exceptional changes in the cell viability and membrane integrity of PBMC after one long day of incubation, and cell viability percentage was similar to untreated cells. However, H_2_O_2_-treated cells (positive control) expressed 69.9 ± 0.18% cytotoxicity, while bionanocomposite treated do not have cytotoxic effects similar to untreated cells; thus indicating they are safe for use as drugs. Further confirmation of safety aspects requires *in vivo* studies to ensure absolute safe usage.

### 3.13. Biocompatibility of the Bionanocomposite

For the drug application and engineering materials, TiO_2_ nanoparticles and their bionanocomposites must be nontoxic and biocompatible. The cytotoxicity of TiO_2_ nanoparticles and their bionanocomposites was evaluated *in vitro* A549 cancer cells. The viability of A549 cells exposed to TiO_2_ nanoparticles and its bionanocomposite with different oil concentrations is presented in Figure 13(a). The results showed that A549 cells can adhere and proliferate on both TiO_2_ nanoparticles and its bionanocomposite. The absorbance of all the samples increases with the increase in culture time, suggesting the well growth of the cells. No visible decrease in viability between TiO_2_ nanoparticles and their bionanocomposites can be noticed at 1, 5, and 10 culture days. Considering the nonsignificant variances (*p* < 0.05) between the investigated samples, bionanocomposite displayed comparable biocompatibility with TiO_2_ nanoparticles. The obtained results were in agreement with previous reports, oil-based polymeric bionanocomposite showed noncytotoxicity to many cells [75], suggesting that bionanocomposite have better cytocompatibility. However, the OD values of TiO_2_ nanoparticles and bionanocomposite were lesser than control (PBS) particularly after 10 days of culture at 570 nm. This can be attributed to the strong hydrophobic character of control compared to TiO_2_ nanoparticles and bionanocomposite; cell adhesion proteins tend to stick to the hydrophobic surface.  Figure 13(b) demonstrates the SEM images of A549 cells after culture at 1, 5, and 10 days on TiO_2_ nanoparticles and bionanocomposite. Fibroblast cells started to express round or fusiform shape on the surface of TiO_2_ nanoparticles and bionanocomposite after immediately 24 h seeding, suggesting that the cells can be easily attached to these nanomaterials. After five-day culture, it was observed that fibroblasts attached to the surface of nanomaterials changed their original shape to fusiform. The proliferation of cells continued on the surfaces of the samples and became subconfluent on the 10^th^ day of the culture. Morphological techniques were applied to further evaluate the phenotype and the interaction of the cells on each sample surface. As shown in SEM images of the 5 days cultured in control, TiO_2_ nanoparticles, and bionanocomposite, the original shape of fibroblasts adhered to all the surfaces changed to fusiform shape. A well-expanded spindle morphology with intercellular tight junctions with nearby cells was observed in cells grown on TiO_2_ nanoparticles and bionanocomposite. However, a slight difference in the cell morphology was noticed in the cells grown on TiO_2_ nanoparticles and bionanocomposite surfaces. More flattened cells on the surface of bionanocomposite were observed in contrast to TiO_2_ nanoparticles, which can be attributed to a much rough surface of the bionanocomposite (Figure 13(b)). Generally, the nanotopography characteristics and surface chemistry are the responsible factors for the cell behavior of the bioactive material. Furthermore, the roughness of bionanocomposite surface and the presence of TiO_2_ nanoparticles on its surface promote the attachment of the cells. Thus, the outcome of the MTT assay and morphological changes confirmed that bionanocomposite is a biocompatible material that can be applied as a future cell culture scaffold.

### 3.14. Photocatalytic Potential of the Bionanocomposite

The photocatalytic effect of bionanocomposite was measured on the basis of the rate of degradation of methylene blue (MB; organic dye pollutant). The MB degradation rate was determined as the percentage of decoloration in contrast to time based at the 660 nm wavelength. The obtained results showed that bionanocomposite expressed a potent photocatalytic effect under UV as well as visible light in contrast to control (Figure 14). The as-synthesized bionanocomposite displayed approximately 7.9 times higher effects than the blank solution used under sunlight.

## 4. Conclusion

A simple, ultrasensitive, and ecofriendly method was developed to fabricate *P. cylindraceus* oil/TiO_2_/PEG bionanocomposite. The fabricated bionanocomposite film was examined using various microscopic and spectroscopic techniques to confirm the well-dispersed *P. cylindraceus oil* and TiO_2_ nanoparticles in the polymeric matrix PEG. The surface morphology of the film showed a well distribution of TiO_2_ nanoparticles with particle size in the range of 60–80 nm. The antibacterial potential of the fabricated film has been screened against four bacterial strains: *S. aureus*, *E. coli*, *P. aeruginosa*, and *S. typhi*. It was observed that the bionanocomposite film exhibited excellent antibacterial activity against *E. coli* and *S. aureus*. The anticancer effect of the fabricated bionanocomposite-film-enriched TiO_2_ nanoparticles also has been evaluated against human lung carcinoma.

## Figures and Tables

**Scheme 1:** Schematic demonstration of (a) TiO_2_ nanoparticles' synthesis using the *P. cylindraceus* aqueous extract and (b) *P. cylindraceus* oil-TiO_2_-PEG bionanocomposite fabrication.

**Figure 1:** GC-MS analysis of *P. cylindraceus* oil.

**Figure 2:** (a) UV-Vis spectrum of TiO2 nanoparticles and (b) average particle size using the particle size analyzer.

**Figure 3:** SEM images of TiO_2_ nanoparticles at (a) 30,000x and (b) 50,000x magnifications.

**Figure 4:** SEM images of (a) PEG, (b) *P. cylindraceus* oil, (c) *P. cylindraceus* oil-PEG, and (d) polymeric *P. cylindraceus* oil-TiO_2_-PEG bionanocomposite.

**Figure 5:** (a) XRD analysis of TiO_2_ nanoparticles synthesized from the *P. cylindraceus* aqueous extract and (b) XRD patterns of (A) plain PEG, (B) *P. cylindraceus* oil-PEG, and (C) polymeric *P. cylindraceus* oil-TiO_2_-PEG bionanocomposite.

**Figure 6:** SEM images of (a) PEG and (b) TiO_2_ nanoparticles dispersed in the polymeric *P. cylindraceus* oil-TiO_2_-PEG bionanocomposite and EDX spectra of (c) PEG and (d) polymeric *P. cylindraceus* oil-TiO_2_-PEG bionanocomposite.

**Figure 7:** Thermogravimetric analysis of *P. cylindraceus* oil/PEG/TiO_2_ bionanocomposite films containing different concentrations of 5, 10, and 15 w% of PEG/TiO_2_ NP.

**Figure 8:** (a) Antibaterial activity of the polymeric *P. cylindraceus* oil-TiO_2_-PEG bionanocomposite against *S. aureus* and *E. coli* and (b) minimum bactericidal concentrations (*μ*g/ml) of the polymeric bionanocomposite against (A) *S. aureus* and (B) *E. coli.* Results are demonstrated as mean ± SD of triplicate experiments.

**Scheme 2:** Schematic representation of the mechanism of antibacterial and cytotoxicity effects of the polymeric *P. cylindraceus* oil-TiO_2_-PEG bionanocomposite.

**Figure 9:** SEM images of untreated and treated with the polymeric bionanocomposite and altered shape of *E. coli* and *S. aureus*.

**Figure 10:** Antiproliferative activity of the polymeric bionanocomposite on A549 cells at 24 h as assessed by the (a) MTT assay to evaluate cytotoxicity, (b) LDH leakage to evaluate membrane integrity, and (c) phase-contrast images demonstrating morphological changes. The arrowheads indicate that the cells have undergone apoptosis exhibiting characteristic features such as shrinkage of the cell, cell density reduction, and production of apoptotic bodies. The data are presented as mean ± SD of triplicate experiments. ^*∗*^*p* < 0.05 expressed the statistically significant differences between the treated groups and control.

**Figure 11:** (a) Fluorescence microscopic images of A549 cells treated with JC-1 staining to assess the mitochondrial membrane potential (ΔΨm) of polymeric bionanocomposite-treated cells after 24 h incubation in contrast to cisplatin (40x); (b) histograms demonstrating the percentage of cells with disrupted MMP; (c) fluorescence microscopic images of CM-H2 DCFDA-treated A549 cells, intracellular ROS indicator after treatment with polymeric bionanocomposite; (d) fluorescence spectroscopy for quantification of the ROS level. Data are displayed as mean ± SD of triplicate measurements.

**Figure 12:** Apoptotic potential of the polymeric bionanocomposite at its IC_50_ in A549 cells as illustrated by (a) AO/EtBr double staining, (b) quantification of apoptotic cells, (c) DAPI staining, and (d) safety assessment of the polymeric bionanocomposite (20–100 *μ*g mL^−1^) on PBMC in comparison with 100 *μ*M H_2_O_2_ after 24 h. Results are expressed as mean ± SD of triplicates, and the values are considered significant at  ^*∗*^*'* ^*∗∗*^*p* < 0.05 treated vs. control.

**Figure 13:** (a) MTT viability assay of A549 cells after 1-, 5-, and 10-day cell culture on PEG and bionanocomposite in comparison to the control (PBS) and (b) SEM images of the fibroblast (A549 cells) on TiO_2_ NPs and bionanocomposite at 1, 5, and 10 days.

**Figure 14:** Photocatalytic activity of the MgO NPs expressed as percentage of methylene blue dye degradation.

**Table 1:** Characterization of essential oil components of the aerial part of *P. cylindraceus*.

S.No	Name of compound	LRI	Area (%)
1	*α*-Thujene	932	0.68
2	*α*-Pinene	935	1.08
3	Camphene	950	2.52
4	Sabinene	975	0.51
5	*β*-Pinene	978	1.52
6	1-Octen-3-ol	980	1.13
7	3-Octanol	988	2.1
8	*β*-Myrcene	993	1.52
10	*α*-Terpinene	1018	3.25
11	p-Cymene	1027	4.82
12	Limonene	1031	1.05
13	**1,8-Cineole**	1036	21.84
14	*γ*-Terpinene	1061	1.82
15	cis-Sabinene hydrate	1069	0.54
16	Linalool	1101	1.72
17	*α*-Thujone	1108	0.85
18	2-Methyl-6-methylene-1,7-octatrien-3-one	1146	0.69
19	**Camphor**	1148	38.85
20	2,6-Dimethyl-1,5,7-octatrien-3-ol	1159	1.89
21	Terpinen-4-ol	1182	2.39
22	*α*-Terpineol	1194	0.82
23	*α*-Copaene	1382	0.4
24	*β*-Caryophyllene	1428	0.18
25	*α*- Humulene	1462	0.62
26	*β*-Selinene	1492	0.44
27	*α*-Bulnesene	1512	0.15
28	*γ*-Cadinene	1521	0.32
29	*α*-Cadinene	1535	0.21
30	cis-Sesquisabinene hydrate	1542	0.12
	Total identified components	96.54	

**Table 2:** Results of hydrolytic degradation of bionanocomposite (90%) film expressed as weight loss (%).

Time (week)	Wight loss % of bionanocomposite (90%)
2	2.75
4	5.7
6	13.54

**Table 3:** Antibacterial activity *P. cylindraceus* oil and *P. cylindraceus* oil/TiO_2_/ PEG bionanocomposite against gram positive and gram negative bacteria.

S. no.	Samples	Concentration (*μ*g mL^−1^)	Antibacterial activity			
			*S. aureus*	*E.coli*	*P. aeruginosa*	*S. typhi*
			Zone of inhibition (mm)	Zone of inhibition (mm)	Zone of inhibition (mm)	Zone of inhibition (mm)
1	*P. cylindraceus* oil	25 50 100	10.08 ± 0.68 10.94 ± 0.64 14.52 ± 0.68	11.08 ± 0.54 12.56 ± 0.56 16.12 ± 1.20	8.83 ± 0.32 9.23 ± 0.24 10.06 ± 0.26	8.25 ± 0.64 9.32 ± 0.62 9.50 ± 0.68
2	*P. cylindraceus* oil /TiO_2_/ PEG bionanocomposite	25 50 100	10.96 ± 0.86 13.28 ± 1.22 20.03 ± 1.20	13.32 ± 1.08 16.42 ± 1.06 25.05 ± 1.08	10.45 ± 0.86 10.93 ± 1.06 12.68 ± 1.04	10.08 ± 1.08 10.92 ± 1.06 11.08 ± 1.08
3	Ciprofloxacin	50	29.15 ± 1.28	39.23 ± 1.28	28.88 ± 1.22	32.25 ± 2.26

**Table 4:** Minimum bactericidal activity of polymeric bionanocomposite against *S. aureus* and *E. coli*.

Sample	CFU mL^−1^	
	*S. aureus*	*E. coli*
Control	TNTC	TNTC
5	TNTC	TNTC
10	TNTC	TNTC
20	TNTC	TNTC
40	TNTC	TNTC
80	TNTC	TNTC
160	2 × 102	4 × 104
320	152	1 × 102
640	3	NIL
1280	1	NIL

## Data Availability

The data used to support the findings of this study are included within the article.
